RETRACTED

# The Application and Evaluation of Effective Quality Management by Objectives in Patient Care for Persistent Vacuum Sealing Drainage

**DOI:** 10.1155/2021/1234003

**Published:** 2021-08-19

**Authors:** Lili Zhao, Jianing Yang, Mingyang Nie, Dan Wang, Guojie Yan, Shuying Li

**Affiliations:** Affiliated Hospital of Chengde Medical University, Chengde City, Hebei Province 067000, China

## Abstract

To investigate the application and evaluation of effective quality management by objectives in patient care for persistent vacuum sealing drainage (VSD), a total of 164 patients with fractures of the hands and feet combined with soft tissue damage admitted to the department of hand and foot surgery in a provincial tertiary hospital from January 2018 to January 2020 were selected as study subjects. The patients were randomly divided into observation and control groups based on the types of fractures, with 82 patients in each group, and both groups underwent VSD surgery for treatment. Both of the groups were cared for VSD using the original nursing model and were compared in terms of treatment compliance, wound recovery, the occurrence of complications, and patient satisfaction with nursing work. The treatment compliance of patients in the observation group was higher than that of the control group (*P* < 0.05). Moreover, the wound healing condition in the observation group and the postoperative wound recovery data were better. The hospitalization time and the number of replacement suckers were less (*P* < 0.05), which met the requirements of statistical research. This confirmed that the application of quality management by objectives in patient care can improve patient compliance with treatment, promote wound healing, reduce the occurrence of corresponding postoperative complications in patients, and improve patient satisfaction with health nursing, which can be promoted for use in the workplace.

## 1. Introduction

The persistent vacuum sealing drainage (VSD) was originally developed by Fleischman et al. [1] and is now more commonly used in patients with fractures combined with soft tissue injuries and makes it an effective clinical treatment [2]. VSD refers to the use of continuous vacuum suction to cover the wound. It allows an easier discharge of the exudate and provides an enhanced clearance effect compared with traditional treatment. The use of a VSD method may completely remove exudate, necrotic fluid, and bacteria from the wound surface via a continuous vacuum, eliminating local dead space, reducing tissue edema, and making granulation tissue easier to grow.

The application of VSD for treatment can reduce the length of hospitalization, reduce the number of dressing changes, and reduce the cost of hospitalization for patients. However, complications may occur when applying VSD for treatment, which can be reduced if the VSD treatment is aided by scientific and rigorous nursing measures. The management by the objective model is a modern management style [3], which emphasizes a goal-oriented, people-centered, and results-based management model, and its application can lead to better results for teams and individuals [4, 5]. Management by objectives in a hospital is a strategic management model that aims to improve the performance of nurses by clearly defining objectives that are agreed to by both management and nurses. Quality management by objectives in patient care is highly correspondent and scientific and has been more widely used in clinical practice in recent years [6, 7]. This study aims to improve the quality of nursing and reduce complications after VSD by setting reasonable quality nursing goals and adopting appropriate nursing measures. A total of 164 patients with fractures of the hands and feet were examined and were compared in terms of treatment compliance, wound recovery, the occurrence of complications, and patient satisfaction with nursing work using management by objective measures. The wound healing condition in the observation group and the postoperative wound recovery data was better, and the hospitalization time and the number of replacement suckers were also less (*P* < 0.05) in the observation group as compared to the control group, which met the requirements of statistical research.

RETRACTED

The rest of this study is organized as follows.  Section 2 provides the detail of the proposed VSD and management by the objective method. The results are presented in Section 3.  Section 4 is about discussion.  Section 5 concludes the study with a summary and future directions.

## 2. Methodology

### 2.1. General Information

A total of 164 patients with fractures of the hands and feet combined with soft tissue damage were admitted to the department of hand and foot surgery in a provincial tertiary hospital from January 2018 to January 2020 were selected as study subjects as given in Table 1. The observation group comprised of 61 males and 21 females, aged 14–70 years, mean age (47.11 ± 14.38) years. Among them, 45 cases were of open hand injuries and 37 cases of open foot injuries. The control group included 69 males and 13 females, aged 12–77 years, with mean age 49.59 ± 14.07 years. In the control group, 45 cases were of open hand injuries and 37 cases of open foot injuries. There was no significant difference (*P* > 0.05) between the two groups comparing the patient data in terms of basic information such as gender, age, and injured part, and the study was approved by the medical ethics committee. The inclusion criteria were as follows: (i) patients willing to voluntarily participate in the study, (ii) patients were diagnosed with fracture combined with soft tissue injury, (iii) the wound area was 4–42 cm^2^, and (iv) the main treatment method was VSD.

RETRACTED

The exclusion criteria were as follows: (i) patients were excluded if the treatment duration was less than 5 days, (ii) patients having mental or cognitive impairment, (iii) patients with chronic diseases, (iv) patients with severe organic lesions in organs, and (v) patients with indications for amputation surgery.

### 2.2. Research Methodology

The surgical methods used in both groups were as follows: preoperative tests were completed in both groups, including blood routine tests, blood group identification, four coagulation tests, two preoperative tests, full biochemical tests, electrocardiogram tests, and culture of wound secretions. The major steps were as follows: (i) remove the necrotic tissue, (ii) cut the VSD dressing according to the size of the wound and apply it to the wound, suture the dressing puncture with the drainage tube, or flow out both the flushing drainage tube and the spare drainage tube, (iii) dry the skin and cover the entire dressing area with a bio-semipermeable membrane to close the wound, (iv) connect the drainage tube to the central negative pressure device, and (v) continuous negative pressure suction for 7–10 d.

#### 2.2.1. Control Group

The control group used the original nursing method. The nurse followed the doctor's advice to implement nursing measures such as drug administration and line nursing, monitored the patient's vital signs and drainage according to the nursing level, observed the changes in the patient's condition, wrote nursing records on time, and improved the patient's basic nursing and postoperative functional exercise instruction.

#### 2.2.2. Observation Group

The observation group used quality management by objectives in the patient care method, which included the following aspects:

- Set goals: the nursing quality goals were established based on the completion of VSD nursing in last 2017, and the nursing pass rate and goal knowledge rate were set as process indicators. The goals and process indicators required all nurses to know and can properly perform their nursing duties and understand how to evaluate and achieve the goals set. The nursing pass rate required nurses to be evaluated and scored according to the VSD nursing evaluation criteria, and 92 points were required to achieve the nursing pass rate; the goal awareness rate required that 100% of all nurses were aware of the VSD nursing quality goals.
- Establish a nursing quality objective management group. The head nurse was the team leader responsible for the overall guidance. Several other key nurses of the department had a different division of labor. The management by objectives team members studied relevant theoretical knowledge, deliberated on the management by objectives process, and developed VSD nursing evaluation criteria. The criteria included the scores of multidimensional evaluations such as maintaining pressure, maintaining confinement, wound nursing, dietary guidance, rehabilitation exercise, psychological nursing, and medication guidance, and nursing of complications ≥92 was considered qualified. Moreover, the nursing quality goal in 2018 was a qualified rate of VSD drainage nursing ≥96%, and the nursing quality goal in 2019 was a qualified rate of VSD drainage nursing ≥97%. In addition, the VSD drainage nursing pass rate was equal to several patients meeting VSD nursing standards/total number of patients treated with VSD × 100%.
- Nursing quality management by objectives implementation measures: nursing quality management provides a comfortable and quiet environment for patients, does basic nursing work, reduces the number of companions, and avoids adverse stimulation. For patients with serious injuries, their treatment period is longer, the hospitalization cost is also usually higher, along with anxiety, psychological nursing is provided by nurses with high seniority to provide preoperative guidance for patients, and personalized guidance according to patients” ages, genders, occupations, and explanation of similar successful surgical cases. The main steps are as follows. (i) Prepare for the operation: the surgeon prepares the surgical instruments, the operating room nurse prepares the operating room, and the department nurse cleans the affected skin and applies antibiotics prophylactically. (ii) Postoperative nursing: postoperative 48 h is the key period of VSD nursing, the patient should be in the supine position, with the affected limb raised with a soft pillow, so that the affected limb is above the heart level and the venous return is not blocked, and the swelling and pain of the injured limb is reduced; adjust the negative pressure value between 0.04 and 0.06 MP according to medical advice. The small pressure does not play the role of drainage, whereas the large pressure leads to wound bleeding. If the VSD dressing collapsed, the flow of fluid in the drainage tube indicates that the wound is well sealed and the negative pressure is effective. If the VSD dressing is swelled and the blood in the drainage tube is dry, the wound is leaking air and the drainage has failed, the drainage bottle is fixed on the floor under the bed using a self-designed fixation bracket. The patient is instructed not to pull, press, or bend the drainage tube when turning over and not to put pressure on the VSD dressing; the bracket can be used to frame the high cover quilt without compressing the surgical part to keep the drainage unobstructed. Nursing staff should patrol patients according to the level of nursing and observe the color, nature, and amount of drainage fluid. The VSD surgery should strictly comply with the principle of aseptic operation and postoperative connection using disposable sterile drainage tubes and vacuum drainage bottles to be used after sterilization; each connection should be tightly connected to ensure the closed sterility of the device, after using the VSD biological semipermeable membrane. It is strictly prohibited to use sharp objects to puncture the semipermeable membrane, thus invalidating the negative pressure. Patients should be encouraged to eat a high-quality protein, calorie-rich, vitamin-rich diet, drink as much water as possible, quit smoking and alcohol, refrain from drinking caffeinated beverages, and refrain from eating stimulating foods such as chili peppers. Patients should perform functional exercises gradually under the guidance of nursing staff, mainly to prevent the occurrence of deep vein thrombosis in the lower limbs; postoperative medications should be used according to medical advice, and the effects and adverse reactions of medications should be observed; patients' general condition and local granulation tissue growth in the wound should be observed, and the sucker and semipermeable membrane were replaced when necessary. (iii) Pain nursing: this ensures that the environment is quiet, so that the patient gets sufficient rest. The patient tries to relax, makes a reasonable assessment of the patient's pain, and applies pain medication as prescribed by the doctor when needed. (iv) Wound nursing: observe the amount of bleeding from the wound and report the drainage to the doctor in charge in a timely manner. Replace the biomembrane after 7 days and observe the growth of granulation tissue on the wound and the color change of the wound. (v) Prevention of complications: the VSD technique is prone to complications such as blockage of drains, the dressing became hard, bleeding, pain, and detachment. The nursing staff should provide all-around health education to patients by making publicity cards, brochures, and minilectures and take individualized instructions for different patients to reduce the occurrence of complications.

RETRACTED

### 2.3. Assessment Methods

The office nurses register the patients included in the study and apply the VSD nursing evaluation criteria to assess the nursing work of the responsible nurses. Moreover, they perform statistical calculations of the pass rate every month, and the head nurse gives appropriate encouragement to the nurses who completed nursing work of higher quality.

### 2.4. Continuous Improvement of Nursing Quality

The management by objectives team summarizes and analyzes the management by objectives work of the previous month at the beginning of each month, and the head nurse identifies the problems that need to be solved by using the Pareto diagram every quarter, and the fishbone diagram to identify the root causes and takes the corresponding nursing measures. They arrange the nursing team meeting to communicate them to every nurse in the department to achieve continuous improvement of nursing quality.

### 2.5. Observation Indicators

- Patients' compliance was recorded in 5 separate assessments of rest, diet, smoking cessation, timely medication administration, and functional exercise. The patients' compliance was further divided into complete compliance where compliance was recorded in all 5 areas, partial compliance where compliance was recorded in 3 areas, and occasional compliance in the other 2 areas; and noncompliance: compliance in less than 3 areas.
- Prognosis of patients in both groups: in this case, the nurses observed the wound reduction, stage II surgery, length of hospitalization, number of dressing changes, and number of sucker changes
- Postoperative complications in both groups: after surgery, the nurses observed and recorded the drainage tube blockage, the dressing became dry and hard, hemorrhage, pain, and tube detached
- Satisfaction with nursing in both groups: A satisfaction survey was conducted before patients are discharged and both satisfied and basic satisfied were classified as satisfied.

### 2.6. Statistical Analysis

The treatment data statistics were recorded using an Excel sheet [8, 9]. The SPSS 23.0 software was applied for data processing, count data were expressed as *n*, and chi-square values were tested. The measurement data were expressed as mean ± standard deviation (*x* ± *s*), the *t*-test was applied, and the percentage compliance rate, incidence rate, and satisfaction were calculated. The *P* < 0.05 was considered statistically significant.

## 3. Results

### 3.1. Comparison of Treatment Compliance between the Two Groups of Patients

The treatment compliance of the observation group was higher than that of the control group, and the difference was statistically significant (*P* < 0.05). The results are given in Table 2. The compliance rates of the observation and control groups were 93.90% and 78.05%, respectively, which show that the compliance rate of the observation group was 15% greater than that of the control group.

RETRACTED

Table 3 represents the wound healing report in both groups. It is evident that, in the observation group, the wound healing condition, the postoperative wound recovery, the hospitalization time, and the number of replacement suckers were all less (*P* < 0.05) than that of the control group. Likewise, the wound area of the observation group was larger, the hospitalization time was shorter, and the number of dressing changes was less, but the difference was not statistically significant (*P* > 0.05).

### 3.2. Comparison of Postoperative Complications between the Two Groups of Patients

The incidence of postoperative complications in the observation group was lower than that in the control group, and the difference was statistically significant (*P* < 0.05), as given in Table 4. The incidence rate of complications in the observation and control groups was 9.76% and 30.49%, respectively. This shows that about a 17% reduction in the incidence rate was reported in the case of the observation group of patients.

### 3.3. Comparison of Patient Satisfaction with Nurses' Work between the Two Groups

Table 5 provides the comparison results for patient's satisfaction with nurses between the observation and control groups. Patient satisfaction in the observation group was higher than that in the control group, and the difference was statistically significant (*P* < 0.05). The satisfaction rate of the observation and control groups reported was 96.34% and 85.37%, respectively. The satisfaction degree of the observation group was about 11% greater than that of the control group.

## 4. Discussion

Soft tissue damage is a common orthopedic injury following open hand and foot injury, and many patients have fractures accompanied by damage to tendons, nerves, and blood vessels, seriously affecting the patient's work and life [10]. The VSD is currently an effective technique for the treatment of refractory and complex wounds, especially in the treatment of soft tissue defects and infected wounds [11, 12]. Since the skin of the hand and foot area is relatively thin, the bones and tendons tend to leak out after injury, and the traditional debridement and dressing procedures tend to cause a secondary infection of the wound, which has a very negative impact on the repair of the patient's wound. Many studies, both domestic and international, have found that VSD negative pressure can affect skin fine vesicles, which can accelerate the secretion of growth factors and accelerate the growth and repair of local skin tissue, which is conducive to the growth and recovery of traumatic vessels in patients. In addition, VSD technology can completely replace the drug exchange treatment method and can reduce the pain of patients and alleviate the economic burden of patients [13].

RETRACTED

Management by objectives theory was developed by Peter Drucker [14]. At its core, Drucker argued is “management by self-control” develops and utilizes the full potential of human beings to mobilize their initiative to achieve the corresponding predetermined goals and continuously improve the quality of nursing. Patients are at the center of nursing quality management to provide higher quality nursing to patients, standards, and processes that are developed, so that members of the organization can coalesce and work towards achieving their goals. Patients with open hand and foot injuries vary greatly in age, injury, literacy, and surgical approach, and individual nursing needs vary, making it necessary to provide individualized nursing to patients.

When quality management by objectives in patient care is applied to the nursing of VSD technology, it can reasonably optimize the configuration of various nursing measures in the perioperative period, which is conducive to improving the nursing staff's nursing ability and also to enabling closer cooperation between medical and nursing [11]. In this way, the occurrence of nursing adverse events can be controlled, the incidence of medical disputes can be reduced, and a good doctor-patient relationship can be maintained by being able to reasonably deal with unexpected situations when they arise, so that the worries and tensions of patients and families can be reduced [12]. We have closely integrated the management by objectives approach with the three aspects of nursing theory and practice to avoid blindness and subjectivity in nursing and to enable homogenization of nursing quality.

VSD technology has high requirements for nursing skills, so a series of nursing measures and evaluation criteria developed by nursing quality management by objectives can ensure that the therapeutic effect of VSD technology is maximized. The workload of medical and nursing staff is reduced, and also, the postoperative complications of patients are effectively reduced. Through management by objectives, the head nurse and nurses jointly determine goals and strengthen the awareness of active participation in nursing safety management. The active execution is enhanced, so that nurses automatically and consciously self-manage according to the content of the goals and complete them on time and with quality^.^ The management by objectives is an effective management method that integrates organizational goals and individual goals and advocates that all people in the organization should work with the same goal to obtain the best results [15]. Through management by objectives, the nurse manager and nurses jointly determine goals, strengthen the awareness of active participation in nursing safety management, and enhance the active execution, so that nurses automatically and consciously self-manage according to the content of the goals and complete them on time and with quality. As this study accomplished the predetermined nursing quality goals, it enhanced the nursing staff's confidence in their work and improved the nurses' sense of achievement in practice to a great extent.

RETRACTED

In this study, a total of 164 patients with fractures of the hands and feet were examined. The patients were divided into observation and control groups. Both of the groups were treated for using the original nursing model. The patients of both groups were compared in terms of treatment compliance, wound recovery progress, complications, and patient satisfaction with nurses. It was observed that the treatment compliance of patients in the observation group was higher than that of the control group (93.90% > 78.05%). Moreover, the wound healing condition in the observation group and the postoperative wound recovery data were better in the observation group. The incidence rate of complications in the observation group was also less than the control group (9.76% > 30.49). This proved that the application of quality management by objectives in patient care can improve patient compliance with treatment, promote wound healing, and reduce the occurrence of corresponding postoperative complications in patients.

## 5. Conclusion

The persistent vacuum sealing drainage is an effective clinical treatment for more patients with fractures combined with soft tissue injuries. The VSD treatment can reduce the length of hospitalization, reduce the number of dressing changes, and reduce the cost of hospitalization for patients. In this study, 164 patients with fractures of the hands and feet were examined. The patients were randomly divided into observation and control groups and both groups underwent VSD surgery for treatment. Both of the groups were cared for and were compared in terms of treatment compliance, wound recovery, the occurrence of complications, and patient satisfaction with nursing work. The treatment compliance of patients' wound healing, recovery, and satisfaction with the nursing group of the observation group was significantly higher than that of the control group, which proved the significance of the proposed research. Although the results of the proposed study are encouraging, the application of quality management by objectives in patient care for VSD needs to be further conducted to confirm its specific clinical role.

RETRACTED

## Figures and Tables

**Table 1:** Comparison of basic conditions between two groups of patients.

Variable		Observation group (*n* = 82)	Control group (*n* = 82)	*t*/2/*U* value	*P* value
Age		47.11 ± 14.37	49.74 ± 14.07	1.186	0.237

Gender	Male	61 (74.4)	69 (84.1)	2.375	0.123
	Female	21 (25.6)	13 (15.9)		

Part	Hand	45 (54.9)	45 (54.9)	0.000	1.000
	Feet	37 (45.1)	37 (45.1)		

**Table 2:** Comparison of treatment adherence between the two groups of patients.

Groups	*n*	Fully compliance	Partially compliance	Noncompliance	Compliance rate (%)
Observation group	82	42	35	5	77 (93.90)
Control group	82	34	30	18	64 (78.05)
*χ* ^2^					8.546
*P*					0.003

**Table 3:** Comparison of prognosis between the two groups of patients (*x* ± *s*).

Groups	*n*	Wound surface reduction	Number of reoperations	Length of hospitalization	Number of dressing changes	Number of replacement suckers
Observation group	82	14.28 ± 8.43	1.43 ± 0.61	15.28 ± 9.98	5.17 ± 4.95	0.04 ± 0.19
Control group	82	13.91 ± 10.88	1.62 ± 0.86	19.12 ± 11.84	6.23 ± 5.05	0.23 ± 0.73
*t* value *(t*值)		0.241	1.682	2.247	1.358	2.358
*P* value (*P*值)		0.810	0.094	0.026	0.176	0.021

**Table 4:** Comparison of postoperative complications between the two groups of patients (cases).

Groups	*n*	Drainage tube blockage	Dressing became dry and hard	Hemorrhage	Pain in the operative area	Tube detached	Incidence rate (%)
Observation group	82	2	2	0	4	0	8 (9.76)
Control group (对照组)	82	6	8	2	8	1	25 (30.49)
*χ* ^2^							10.964
*P*							0.001

**Table 5:** Comparison of patient satisfaction between the two groups (cases).

Groups	*n*	Satisfied	Basic satisfied	Dissatisfied	Satisfaction degree (%)
Observation group	82	46	33	3	79 (96.34)
Control group	82	32	38	12	70 (85.37)
*χ* ^2^					5.944
*P*					0.015

## Data Availability

The data used to support the findings of this study are included within the article.
